# Factors Associated with Utilization of Sexual and Reproductive Health Services among the Youth in Lira City West, Northern Uganda: A Cross-Sectional Study

**DOI:** 10.1155/2023/9649792

**Published:** 2023-05-18

**Authors:** Tom Murungi, Deo Benyumiza, Juliet Apio, Catherine Nekesa, Aisha Nalubuuka, Ivan Misuk, Edward Kumakech

**Affiliations:** ^1^Department of Midwifery, Faculty of Nursing and Midwifery, Lira University, P.O BOX 1035, Lira, Uganda; ^2^Department of Nursing, Faculty of Nursing and Midwifery, Lira University, P.O BOX.1035, Lira, Uganda

## Abstract

**Background:**

The youth in Uganda, as in much of sub-Saharan Africa, face numerous sexual and reproductive health (SRH) challenges, from human immunodeficiency virus HIV infection, and unsafe abortions to unwanted pregnancies. This study, therefore, assessed the utilization of sexual and reproductive health services and associated factors among the youth in Lira city west, northern Uganda.

**Methods:**

This was a cross-sectional study conducted in January 2023 among 386 young people (15-24 years) in Lira city west division, Lira city. Multistage cluster sampling technique was used to recruit our study participants. Data were collected using an interviewer-administered questionnaire. Data were analyzed using SPSS version 23, descriptive statistics, cross-tabulation, bivariate, and multivariate logistic regression analyses. All variables were set by *p* values less than 0.05 and reported adjusted odds ratio with its 95% confidence interval.

**Results:**

The utilization of SRH services was 42.0% (162/386) among the study participants. Family planning, voluntary HIV counseling and testing (VCT), and general counseling services were the most utilized SRH services in the past 12 months. Young people who were aware of SRH services (AOR: 0.24; 95% CI: 0.08-0.74), were aware of a reproductive health facility (AOR, 4.24; 95% CI: 1.62-11.09), discussed SRH issues with peers/friends (AOR, 3.98; 95% CI: 1.53-10.33), had a sexual partner (AOR, 10.00; 95% CI: 4.05-24.69), had sexual intercourse (AOR, 4.59; 95% CI: 2.18-9.69), and had access to SRH services (AOR, 2.68; 95% CI: 1.12-6.40) were more likely to utilize SRH services compared to their counterparts.

**Conclusion:**

This study showed a low utilization of sexual and reproductive health services among youth in Lira city west, northern Uganda. Being aware of SRH services, awareness of reproductive health facilities, discussing SRH issues with peers, having sexual intercourse, having a sexual partner, and access to SRH services were independently associated with the utilization of SRH services. Therefore, there is a need to strengthen sustainable multisector approaches aimed at improving awareness and access to sexual and reproductive health services among the youth.

## 1. Background

Globally, 21 million pregnancies are occurring among adolescents each year, of which 50% are unintended [1]. HIV/AIDS has affected more than half of the world's population that is below 25 years [2]. In addition, the AIDS epidemic remains the leading cause of death among young people aged 10-24 years in Africa [3]. Uganda's young population is 52% of the population, and this is the age that is most affected by HIV/AIDs [2]. Adolescent women aged 15-19 years make up approximately one-quarter of the female population in Uganda, and this age group accounts for 14% of all births [4]. Half of the pregnancies among adolescents in Uganda are unintended, of which 30% end up in abortions [5]. In low and middle-income countries, out of the 32 million adolescent women who want to avoid pregnancy, 14 million have an unmet need for modern contraception [1].

The youth in Uganda, as in much of sub-Saharan Africa, face numerous sexual and reproductive health (SRH) challenges, from HIV infection, and unsafe abortions to unwanted pregnancy [6, 7]. Even those able to find accurate information about their health and rights may be unable to access the services needed to protect their health [8]. Yet, these adolescents are most vulnerable to a range of reproductive health problems, such as teenage pregnancy and childbearing, unsafe abortion, and sexually transmitted infections (STI), including HIV [9]. Hence, adolescents' sexual and reproductive health must be supported by providing access to comprehensive sexuality education; services to prevent, diagnose and treat STIs; and counseling on family planning. In addition, young people need to be empowered to know and exercise their rights—including the right to delay marriage and the right to refuse unwanted sexual advances [8].

The Ugandan government in 2017 has since committed to improving access to contraception for adolescents by implementing the National Adolescent Health Policy and the National Sexuality Education Framework [10]. Consequently, increased investment is essential to ensure that adolescents have access to the age-appropriate information and services they need to determine whether and when to become pregnant. Improving adolescents' sexual and reproductive health and rights, including preventing unintended pregnancy, is essential to their social and economic well-being.

Despite a concerted effort to introduce and scale up adolescent and youth sexual reproductive health (AYSRH), there is a dearth of evidence that suggests low uptake of sexual and reproductive health services among young people [11–13]. Previous studies have shown the barriers to the utilization of sexual and reproductive health services to be having a negative perception of counseling and reproductive health services and about youth-friendly service providers, a lack of knowledge on the advantages of the services, long queues, and inconvenient location of health facilities, among others [12–14]. Other factors include education level, old age of adolescents, out-of-school youth, sex, partner discussion about reproductive health issues, and discussion of reproductive issues with a family member or peers, among others [15–17].

Lira District in northern Uganda reported the highest rate of teenage pregnancy in northern Uganda [18]. In the financial year that ended, 2018/2019, the district recorded 9,916 teenage pregnancies, up from 5,178 in the financial year 2017/2018, and at least 5000 teenagers are impregnated every year [19]. This signifies the unmet need for sexual and reproductive health services in this area. And few studies have been done in this area to assess the level of utilization of sexual and reproductive health services in Lira city. Hence, this study assessed the utilization of sexual and reproductive health services and associated factors among the youth in Lira city west, northern Uganda.

## 2. Materials and Methods

### 2.1. Study Design and Setting

A cross-sectional study with quantitative methods of data collection was conducted in January 2023. The study was conducted among youth aged 15-24 years in the subcounties of Ojwina, Adyel, and Lira. These three subcounties are all found in Lira city west division, Lira city, northern Uganda. Lira city is about 337 kilometers (209 mi), by road, north of Kampala, the capital city of Uganda. Lira city is host to both governmental and nongovernmental organizations working along with health centers and hospitals to provide sexual and reproductive health services to the young population. The services offered by these entities range from awareness creation of SRH, HIV testing, family planning, postabortion care, STI screening, and vaccination services against infectious diseases.

### 2.2. Study Population

This study was conducted among 386 youth aged between 15 and 24 years selected following a multi-stage sampling technique in Lira city west, northern Uganda.

### 2.3. Selection Criteria

#### 2.3.1. Inclusion Criteria

All youth aged 15-24 years residing in Lira city west during data collection time and consented to their participation were enrolled in this study.

#### 2.3.2. Exclusion Criteria

Youths aged 15-24 years, residing in Lira city west during the period of data collection, who were in boarding schools, in a hurry to reach school in time, and those who were working outside Lira city west were excluded from this study.

### 2.4. Study Variables

#### 2.4.1. Dependent Variable

Dependent variable includes the level of utilization of sexual and reproductive services among the youth aged 15-24 years in Lira city west, northern Uganda.

#### 2.4.2. Independent Variable

Independent variables will include social demographic, individual, and health system factors affecting the utilization of sexual and reproductive health services among the youth. These factors included ever-discussed SRH issues, educational level, knowledge of the place of care for family planning services, access to SRH information, having a sexual partner, and ever had sexual intercourse in the past twelve months.

### 2.5. Sample Size Estimation

The sample size was calculated using Kish Leslie's formula (1965) for sample size calculation.

Based on the assumptions that the proportion of the youth who used the sexual and reproductive health services was 50% (*p* = 0.5), the proportion (*q*) who did not use sexual and reproductive health services (*q* = 1 − *p*), and margin of error (*d* = 0.05) and *z* is the standard normal deviation corresponding to 95% confidence level (*z* = 1.96).

(1) $$\begin{array}{c} n=\frac{z^{2}pq}{d^{2}}. \end{array}$$

Hence, considering the 5% nonresponses, our sample size was 422.

### 2.6. Data Collection Method and Tool

We used researcher-administered questionnaires to collect data. The questionnaire was developed from a literature review of previous studies [12, 14, 17, 20] by the research team, reviewed, and adjusted accordingly to fit our study objectives before the actual data collection process. The questionnaire collected information on the following: demographic characteristics of participants (age, marital status, tribe, religion, education level, and staying with parents), utilization of SRH services, individual characteristics (awareness of SRH services, awareness of any SRH health facility, discussion of SRH issues, and having sexual intercourse), and health system factors (access to SRH services, provider recommendation, health worker attitude, and waiting hours at the facility).

### 2.7. Sampling Procedure

The study participants were selected using a multistage sampling technique. Lira city west consists of 3 subcounties (Figure 1). At stage one, out of the 3 subcounties, one was selected randomly. Then, 2 wards from the selected subcounty were selected using a simple random sampling method. Then, from the selected wards, 3 cells were selected from each ward using a simple random sampling technique. Finally, the young people (with an age range of 15 to 24 years) were selected consecutively following their availability. In each household, one young person was asked to participate in the study, and data was collected in 14 days, as shown in the following illustration.

### 2.8. Operational Definitions

*Subcounty:* this is an administrative unit made up of several wards/parishes. A collection of subcounties makes up a county.

*Ward/parish:* this is an administrative unit made up of cells/villages. A collection of wards/parishes makes up a subcounty.

*Cell/village:* this is the lowest administrative unit, and it consists of households.

*“O” level/ordinary level education:* this is the first/lower level in secondary education and runs for four years.

*“A” level/advanced level of education:* this is the second/and upper level of secondary education and runs for two years.

### 2.9. Data Management

The study tools were checked for completeness and consistency after each day of data collection. A data entry screen was created in Microsoft Excel, and data was double entered. Cleaning involved the exclusion of data that was found inconsistent. The data in hard copies were kept under lock and key, whereas data in soft copies were kept on a hard drive only accessible to the investigators.

### 2.10. Data Analysis

Data was exported to SPSS version 23.0 for analysis. Descriptive statistics were used to describe the study population through relevant variables such as sociodemographic characteristics (age, level of education, religion, and marital status). At the univariate level, data were summarized in percentages, proportions, and frequencies, and it enabled us to determine the level of utilization. Bivariate and multivariable models were run to assess any relationship between each independent variable (sociodemographic characteristics, health system, and individual factors) and the outcome variable (young people's sexual and reproductive health service utilization, i.e., at least once SRH service used in 12 months). Crude and adjusted odds ratios were used to ascertain any associations between the dependent and independent variables, while significance was determined using 95% confidence intervals. Independent variables found to be significant with a *p* value less than 0.05 at the bivariate level were included in a multivariable logistic regression model for the dependent variable to control potential confounding variables. The multivariate analysis enabled the researchers to come up with a final model of predictors of SRH utilization.

### 2.11. Ethical Consideration

Ethical approval was obtained from the Gulu University Research Ethics Committee (GUREC-2022-269) and, thereafter, from the town clerk of Lira city before conducting the study. Written informed consent was obtained after providing consent forms to all participants stating the terms and conditions of the study which they are meant to understand before being recruited into the study. Also, assent was obtained from parents of minors, that is to say, youth below 18 years of age. The researchers used unique identifiers instead of the real names of participants to ensure confidentiality. Furthermore, participants were assured that their information is not going to be discussed with any other person.

## 3. Results

### 3.1. Sociodemographic Characteristics of Youth Aged 15-24 Years in Lira City West, Northern Uganda (*n* = 386)

Out of 422 youth, 386 participated obtaining a response rate of 91.5%. Half, 195 (50.5%), of the respondents were females, and most, 262 (67.9%), were in the age group of 20-24 years. In regards to marital status, three-quarters of 277 (71.8%) of the respondents were single. Nearly one-third, 141 (36.5%), of the respondents had completed an advanced level of education, and the majority, 235 (60.9), were living with their parents or relatives (Table 1).

### 3.2. Level of the Utilization of Sexual and Reproductive Health Services among Youth Aged 15-24 Years in Lira City West, Northern Uganda

Out of 386 respondents, more than a third, 162 (42.0%), had ever utilized sexual and reproductive health services in the last 12 months (Figure 2).

In this study, 79(50.0%) had used family planning, 80(50.6%) had used voluntary counseling and testing, 25(6.5%) had used antenatal care services, 44(27.8%) had used sexually transmitted disease diagnosis and treatment, 55(34.8%) had used general counseling services, few 8(5.1%) had used postabortion care services, and very few, 6(3.8%) had used safe abortion in the past 12 months (Figure 3).

### 3.3. Factors Associated with the Utilization of Sexual and Reproductive Health Services among Youth Aged 15-24 Years, in Lira City West, Northern Uganda

In binary logistic regression, the factors that were statistically associated with the utilization of SRH services at *p* value <0.05 were being aware of SRH services (*p* ≤ 0.001), being aware of any reproductive health facility (*p* < 0.001), ever discussing SRH issues with peers/friends (*p* < 0.001), ever having a sexual partner (*p* ≤ 0.001), ever having sexual intercourse (*p* < 0.001), ever participating in peer education (*p* = 0.012), feeling embarrassed while seeking SRH services (*p* = 0.011), ability to access SRH services (*p* < 0.001), judgmental attitude of service providers (*p* = 0.021), and long waiting hours at the SRH clinics (*p* = 0.014). Those which were not statistically significant with the utilization of SRH services were the discussion of SRH issues with parents (*p* = 0.118), ever received sex education (*p* = 0.147), fear of being seen by parents while seeking SRH services (*p* = 0.303), lack of privacy and confidentiality (*p* = 0.220), and the unwelcoming attitude of health workers (*p* = 0.499).

In the multivariate logistic regression model, the factors that were independently associated with the utilization of SRH services among youth aged 15-24 years who were aware of SRH services (AOR: 0.24; 95% CI: 0.08-0.74), being aware of a reproductive health facility (AOR, 4.24; 95% CI: 1.62-11.09), discussion of SRH issues with peers/friends (AOR, 3.98; 95% CI: 1.53-10.33), having a sexual partner (AOR, 10.00; 95% CI: 4.05-24.69), having sexual intercourse (AOR, 4.59; 95% CI: 2.18-9.69), and access to SRH services (AOR, 2.68; 95% CI: 1.12-6.40) were more likely to utilize SRH services compared to their counterparts (Table 2).

## 4. Discussion

Understanding the factors affecting SRH service utilization is pivotal to the attainment of good health for all, especially in northern Uganda where the youth face radical SRH challenges. Findings from this study indicate that less than half (42.0%) of the youth in Lira city west had utilized sexual and reproductive health services. Family planning, voluntary counseling, testing services, and general counseling were the most utilized SRH services in the past 12 months.

This study showed that only 42.0% of the youth had utilized any sexual and reproductive health services in the past 12 months. This finding differs from those obtained in Kampala and Amudat at 61.99% and 66.7%, respectively [12, 17]. This difference could be attributed to variations in awareness, accessibility, and sociodemographic characteristics of participants from both studies. A similar finding was obtained from a study done among young people in the Awabel district, Northwest Ethiopia, 41.2%, [16]. However, this finding was greater than that from the previous studies conducted in Bahir Dar University, 32%, Hadiya zone, 29.4%, and Debre Tabor Town, 28.8%, in Ethiopia [11, 13, 21]. This could also be due to sociocultural variations and differences in service provision and accessibility. Consequently, this contributed to the low utilization of SRH services among the youth in these studies; for instance, Bahir Dar University used traditional reproductive health services because the services which were provided by the health facilities were inconvenient [21]. In addition, despite reporting good SRH awareness, the youth from Debre Tabor Town [13] and Hadiya zone [11] reported unwelcoming attitudes toward health providers and poor access to SRH services they needed, respectively.

Family planning, VCT, and general counseling services were the most utilized SRH services. Comparably, a study among street youth in Kampala showed that 18.13% had used contraception/family planning, and 58.67% had tested for human immunodeficiency virus (HIV) and knew their status [12]. This finding is also consistent with those from previous studies in Ethiopia [20, 22]. This could be justified by the mass availability of family planning services and many testing opportunities in the area which the youth can utilize. This is supported by the fact that Uganda is committed to scaling up the use of modern family planning methods to ensure that every Ugandan woman can choose when and how many children to have [23].

Safe abortion (3.8%) and postabortion care services (5.1%) were the least utilized services. This finding somewhat goes in line with the finding in Nekemte town, Ethiopia [22]. On the contrary, findings from Addis Ababa (59.4%) and Gondar (55.5%) in Ethiopia revealed higher utilization of safe abortion services [24, 25]. However, these studies mainly focused on street children aged 10-18 and 10-24 years old, respectively, which could be responsible for this variation [24, 25]. This finding suggests that many youths could be opting for unsafe options and traditional birth attendants for these services. Evidence in Uganda suggests that women are unable to utilize safe abortion and postabortion care services due to unaffordability accredited to the high costs incurred in a hospital compared to traditional birth attendants [26].

The youth who were aware of sexual and reproductive health services were more likely to utilize them compared to their counterparts. This could be explained by the fact that most youths discussed SRH issues with their peers which could have been a useful source of information for them. This finding is consistent with those from Lagos in Nigeria [27] and eastern Ethiopia [14] where knowledge about SRH was a strong predictor of SRH utilization. Evidence from previous studies suggests that a lack of awareness of some aspects of SRH is responsible for the low uptake of SRH services among the youth [28, 29]. This indicates the need to provide comprehensive knowledge about SRH among the youth to improve utilization.

Participants who were aware of any reproductive health facility were 4.24 times more likely to utilize SRH services than their counterparts. The same results were obtained from studies in Kampala and Ethiopia [12, 13]. This could be accredited to the fact that those who know the reproductive health facilities are well informed about the services offered and know where to access these services leading to utilization. On the other hand, a lack of awareness of where to seek SRH services and the perceived stigma of seeking SRH services from a reproductive health clinic may deter SRH utilization among the youth [30].

Furthermore, young people who discussed SRH issues with their peers and friends were 3.98 times more likely to use SRH services compared to those who did not. This might be due to prior sharing of experiences and opportunities on SRH among the youth hence increasing utilization. This finding conforms with the findings from studies in Ethiopia [31]. However, participants in this study did not prefer discussing SRH issues with their parents as opposed to findings from a study in the Nakivaale refugee settlement in Uganda where the youth discussed their reproductive health concerns with their parents [32]. The variation could be due to the differences in the sociodemographic characteristics of the participants between both studies since the aforementioned study was conducted among the youth in a refugee settlement. Hence, this calls for the development of interventions to strengthen the communication links between parents and youth in areas regarding reproductive health [33]. This is vital in informing the youth about the risk and protective strategies, which is critical in the reduction of risky sexual behaviors [34].

Concerning sexual behavior, those who ever had a sexual partner were 10.00 times more likely to utilize SRH services compared to [13] their counterparts. Similarly, a previous study in eastern Ethiopia supported the same claim [20]. This might be due to sexual partners having discussions on SRH issues and plans of protection before intercourse. In addition, as a way of finding solutions to their sexual and reproductive health problems, thus, they are likely to utilize SRH services. In addition, this study found out that the youth who had ever had sexual intercourse was 4.59 times more likely to utilize SRH services than their counterparts. Likewise, previous studies have shown that having sexual intercourse and being sexually active predict the utilization of SRH services [11, 13, 20, 35]. This could be due to the perceived risk of having unintended or negative sexual outcomes related to engaging in sexual intercourse.

The youth who were able to access SRH services were 2.68 times more likely to utilize these services compared to their counterparts. Comparably, similar findings were obtained from Ethiopia and Nigeria. This could be attributed to easy availability and awareness about SRH services and where to seek them. As a result, young people are motivated to use SRH services. Moreover, evidence from rural Uganda showed that limited access to adolescent and youth-friendly services is responsible for the low utilization of SRH services [17]. Hence, strengthening the implementation of the national guidelines on adolescent sexual and reproductive health could scale the number of youths who can access SRH services they need for their health.

### 4.1. Study Limitations

Due to the cross-sectional nature of this study, it was difficult to establish a causal relationship between the dependent and independent variables. Some of the interview questions required responses from the past which could have potentially introduced recall bias. The study used a self-report instrument which could result in social desirability bias.

## 5. Conclusion

This study showed a low (42.0%) utilization of sexual and reproductive health services among youth in Lira city west, northern Uganda. Family planning, voluntary HIV counseling and testing, and general counseling services were the most utilized SRH services. Predictors for utilization of SRH services were awareness of SRH services, awareness of reproductive health facilities, discussion of SRH issues with peers, having sexual intercourse, having a sexual partner, and access to SRH services. Therefore, there is a need to strengthen sustainable multisector approaches aimed at improving awareness and access to sexual and reproductive health services among the youth.

## Figures and Tables

**Figure 1:** Procedure of multistage sampling.

**Figure 2:** Showing the level of utilization of sexual and reproductive health services among youth aged 15-24 years in Lira city west, northern Uganda.

**Figure 3:** Sexual and reproductive health services used by the youth (15-24 years) in the last 12 months, in Lira city west, northern Uganda.

**Table 1:** Sociodemographic characteristics of youth aged 15-24 years in Lira city west, northern Uganda (*n* = 386).

Variable	Frequency (*n*)	Percentage (%)
Age		
15-19	124	32.1
20-24	262	67.9
Sex		
Female	195	50.5
Male	191	49.5
Marital status		
Single	277	71.8
Cohabiting	71	18.4
Married	38	9.8
Level of education		
No formal education	19	4.9
Completed primary level	55	14.2
Completed “O” level	103	26.7
Completed “A” level	141	36.5
Completed tertiary level	68	17.6
Who do you live with?		
Alone	84	21.8
Parents/relatives	235	60.9
Friends/spouse	67	17.4

**Table 2:** Multivariate analysis of factors associated with the utilization of sexual and reproductive health services among youth aged 15-24 years in Lira city west, northern Uganda.

Variables (*n* = 386)	SRH utilization		COR (95% C.I.)	AOR (95% C.I.)	*p*-value
	No (*n* (%))	Yes (*n* (%))			
Aware of youth SRH services					0.013^∗^
No	59 (15.3)	12 (3.1)	1.00	1.00	
Yes	165 (42.7)	150 (38.9)	4.47 (2.31-8.64)	0.24 (0.08-0.74)	
Aware of any RH facility					0.003^∗∗^
No	72 (18.7)	14 (3.6)	1.00	1.00	
Yes	152 (39.4)	148 (38.3)	5.01 (2.71-9.27)	4.24 (1.62-11.09)	
Discuss SRH issues with peers					0.005^∗∗^
No	51 (13.2)	15(3.9)	1.00	1.00	
Yes	173 (44.8)	147 (38.1)	2.89 (1.56-5.35)	3.98 (1.53-10.33)	
Ever had a sexual partner					≤0.001^∗∗∗^
No	125 (32.4)	10 (2.6)	1.00	1.00	
Yes	99 (25.6)	152 (39.4)	19.19 (9.61-38.34)	10.0 (4.05-24.69)	
Ever had sexual intercourse					≤0.001^∗∗∗^
No	175 (45.3)	39 (10.1)	1.00	1.00	
Yes	49 (12.7)	123 (31.9)	19.19 (9.61-38.34)	4.59 (2.18-9.69)	
Able to access SRH services					0.026^∗^
No	65 (16.8)	14 (3.6)	1.00	1.00	
Yes	159 (41.2)	148 (38.3)	4.32 (2.33-8.03)	2.68(1.12-6.40)	

Level of significance ^∗^*p* < 0.05, ^∗∗^*p* < 0.01, ^∗∗∗^*p* ≤ 0.001, COR: crude odds ratio; AOR: adjusted odds ratio, at 95% confidence interval.

## Data Availability

The data sets used and/or analyzed during the study are available from the corresponding author on reasonable request.
